# Effect and Role of miR-196b in Ectopic Pregnancy

**DOI:** 10.1155/2022/7797484

**Published:** 2022-02-28

**Authors:** Shan Deng, Xiaofeng Su, Xiaoling Li, Xiaomiao Shen, Shengru Chen, Xiaoman Lin, Mushi Ye

**Affiliations:** ^1^Department of Gynaecology and Obstetrics, The Second Affiliated Hospital of Guangdong Medical University, Zhanjiang 524000, Guangdong, China; ^2^Department of Urological Surgery, The Affiliated Hospital of Guangdong Medical University, Zhanjiang 524000, Guangdong, China

## Abstract

Ectopic pregnancy (EP) is associated with significant morbidity and mortality, but the molecular mechanism of this condition is still unclear. miR-196b, a hot research direction for the past few years, participates in the occurrence of various diseases but whether it plays a regulatory role in EP is still unclear. This research was set to investigate the expression and potential value of miR-196b in EP. qRT-PCR was utilized to determine the relative expression of miR-196b in peripheral blood of EP patients and to observe the expression changes of miR-196b before and after treatment. Correlation analysis of miR-196b with HCG and progesterone was performed. Logistic regression analysis was applied to independent risk factors affecting EP patients. TargetScan was utilized to predict the downstream target genes of miR-196b, and GO and KEGG analysis was carried out using the R language pack. qRT-PCR showed that miR-196b expression in peripheral blood of EP patients was lower than that of normal people. miR-196b expression in patients after treatment was notably higher than that before treatment. In addition, correlation analysis showed that miR-196b was positively correlated with the expression of HCG, progesterone, and estradiol. Risk factor analysis revealed that abortion history, pelvic inflammatory disease history, lower abdominal surgery history, and miR-196b were independent risk factors for EP, and the AUC of the combined ROC curve was 0.899. GO function enrichment and KEGG signal pathway enrichment found 10 potential functions and 2 potential signal pathways of miR-196b. miR-196b is expressed in EP patients, is differentially expressed according to the change in EP condition, and is expected to become a promising index for clinical diagnosis of EP.

## 1. Introduction

Pregnancy is a unique clinical situation as it can be accompanied by special diseases [1]. Ectopic pregnancy (EP) is a complication of early pregnancy, in which the fertilized eggs are planted anywhere outside the uterine cavity without entering the uterus. Fallopian tube EP is the most common clinically [2]. At present, the clinical diagnosis of EP is mainly made by ultrasound combined with serum human chorionic gonadotropin (hCG)/progestogen [3]. However, with continuous serum hCG measurement, the patient is at risk of tubal rupture during the delay before the next hCG assessment [4]. In addition, the use of serum hCG and/or progesterone to determine EP is limited by false negative and false positive rates [5]. Hence, we hope to find new potential markers of early EP to solve this problem.

MicroRNAs (miRs) are short-chain noncoding RNAs with a length of 17–21 nt [6]. miRs are used to be able to target downstream genes through the 3-UTR end to regulate cell proliferation, differentiation, and programmed cell death [7, 8]. A close relationship between miRs and EP has been found by more and more studies. For example, the team of Zhang [9] explored the clinical significant of hsa-miR-1247 and hsa-miR-1269a expression in EP caused by salpingitis. miR-196b, as an early discovered miR [10], is differentially expressed in tumors [11]. miR-196b has low expression in EP [12], but in EP it remains unclear. EP is a complication of early pregnancy, and most patients will suffer from severe pelvic pain [13]. At present, the pathogenesis of EP is still unclear. Some scholars believe that embryo retention may be caused by damage to the embryo-fallopian tube environment, which leads to fallopian tube implantation [14, 15].

Hence, we hope to provide potential observation indicators for clinical diagnosis and prognosis judgment through exploring the clinical value of miR-196b in EP.

## 2. Methods and Data

### 2.1. Clinical Data

89 EP patients treated in our hospital from January 2017 to January 2020 were included in the observation group (OG), and 70 healthy pregnant women who underwent physical examination during the same period were included in the control group (CG). The inclusion criteria of EP patients include the following: patients showed symptoms of vaginal bleeding and abdominal pain in the early pregnancy and were diagnosed as EP by ultrasound examination. All the patients in the OG were tubal EP patients. Exclusion criteria include the following: hypertension, salpingitis, preeclampsia, diabetes, mental disorders, or communication disorders, previous surgical treatment, or patients who did not cooperate with the treatment.

### 2.2. Sources of Drugs

The supplier of methotrexate for injection (Item No. H20043647) is Neijiang Huiyu Pharmaceutical Co., Ltd., Sichuan Province. The supplier of Mifepristone (Item No. H10950170) is Zhejiang Taizhou Xianju Pharmaceutical Co., Ltd., China.

### 2.3. Treatment Methods

Patients in the OG were treated with methotrexate combined with mifepristone as follows: patients were injected with a single intramuscular injection of 50 mg/m2. On this basis, mifepristone was orally administered to patients on an empty stomach starting in the morning, with a dose of 75 mg, 6 days a course of treatment, and 2 courses of treatment in total. If patients failed in the treatment process, surgical treatment would be conducted on them.

### 2.4. Detection of HCG and Progesterone

Samples of patients after two courses of treatment were collected. All hCG and progesterone measurements were performed in our hospital using commercially available analysis methods. Serum hCG was determined by Sagittarius total human chorionic gonadotropin (HCG) method and serum progesterone by Centaur Total HCG method.

### 2.5. qRT-PCR

Serum of patients before treatment and after 2 courses of treatment was collected to extract the total RNA using TRIzol kit. Detection of purity, concentration, and integrity of the extracted total RNA was conducted using UV spectrophotometer and agarose gel electrophoresis. Trans Script® miRNA RT Enzyme Mix and 2×TS miRNA Reaction Mix (TransGen Biotech) were applied for total RNA reverse transcription. The procedures were strictly in the light of the manufacturer's kit. Subsequently, PCR amplification experiments were performed. The amplification conditions and amplification system were carried out according to the kit instructions. Three replicate wells were set up for each sample, and the experiment was performed three times. In this study, U6 was taken as an internal reference, and 2-^△△^Ct was utilized to analyze the data [16].

### 2.6. Curative Effect Evaluation

The curative effect of the patients after treatment was evaluated and divided into markedly effective, effective, and ineffective. EP-related symptoms of markedly effective patients were alleviated after treatment. Effective patients had a small amount of vaginal bleeding and abdominal pain after treatment. None of the above conditions were achieved in the ineffective patients.

### 2.7. Functional Prediction of Mir-196b

TargetScan (http://www.targetscan.org/vert_72/) was adopted for prediction of miR-196b target genes, and R language pack was used to enrich GO and KEGG for the predicted target genes to find the potential mechanism of miR-196b.

### 2.8. Statistical Analysis

The GraphPad 8 software package was utilized to draw the required images and analyze the data. Mean ± standard deviation (Mean ± SD) was used for measurement data conforming to normal distribution, and independent sample *t*-test was applied for comparison between groups. The data that did not conform to the normal distribution were expressed as quartiles [Mean (P25∼P75)]. Counting data were expressed by percentage (%); the chi-square test was adopted and expressed by c2. Comparison among multiple groups was made by a one-way analysis of variance. LSD-t test was applied for post-event pairwise comparison. Pearson test was utilized for analysis of the correlation of miR-196b with HCG and progesterone. Logistic regression was applied to analyze the risk factors of miR-196b in EP. Receiver operation characteristic (ROC) analysis was used to draw the area under the curve (AUC) of multivariate meaningful index. When *P* < 0.05, there was statistical difference.

## 3. Results

### 3.1. Comparison of Baseline Data of Patients

First of all, we compared the baseline data between the OG and the CG. Through analysis, we found that there was no statistical difference between the two groups in age, number of pregnancies, smoking history, place of residence, and nation (*P* > 0.05), while the concentration levels of HCG, progesterone, and estradiol in the OG were considerably lower than those in the CG, with a statistical difference (*P* < 0.001), as shown in Table 1.

### 3.2. Expression of miR-196b in EP Patients and Its Correlation with HCG and Progesterone

In order to measure the expression of miR-196b in EP patients, we detected it in patients' peripheral blood by qRT-PCR. Through analysis, we found that it decreased in EP patients. We further analyzed the relationship of miR-196b with HCG and progesterone and found that miR-196b was positively correlated with the expression of HCG, progesterone, and estradiol, suggesting that miR-196b may be a promising marker for diagnosing EP (Figure 1).

### 3.3. Changes of miR-196b in EP Patients before and after Treatment and Its Expression in Patients with Different Curative Effects

In the above study, we determined that miR-196b expressed highly in EP patients, but whether miR-196b expression changes after treatment in EP patients is unclear. Therefore, we treated EP patients with methotrexate combined with mifepristone, such as 40 patients with markedly effective efficacy, 39 patients with effective efficacy, and 10 patients with ineffective efficacy. Patients' peripheral blood was collected and analyzed; the results showed that miR-196b expression was higher after treatment than before treatment. In addition, miR-196b expression in peripheral blood gradually increased as patients improved, which suggested that miR-196b can be used as a potential indicator to observe the curative effect of EP patients after treatment as shown in Figure 2.

### 3.4. Analysis of Risk Factors for EP Patients

In this study, we also analyzed the risk factors for EP. First, we conducted univariate analysis and found that pelvic inflammatory disease history, lower abdominal surgery history, abortion history, and miR-196b were risk factors for EP in the OG. Further, multivariate analysis revealed that abortion history, pelvic inflammatory disease history, lower abdominal surgery history, and miR-196b were independent risk factors of EP. Furthermore, we drew the joint ROC curve according to the indicators with different factors and found that abortion history, pelvic inflammatory disease history, lower abdominal surgery history, and miR-196b had certain clinical value in the diagnosis of EP, as shown in Tables 2 and 3and Figure 3.

### 3.5. miR-196b Functional Analysis

Here, we determined the clinical value of miR-196b in EP, but we did not carry out relevant basic research to further analyze the role of miR-196b. Hence, we analyzed the promising target genes of miR-196b to pave the way for our subsequent research. We predicted the target genes of miR-196b by TargetScan and found 356 potential target genes. Then, we annotated the target gene with GeneID using org.Hs.eg.db package in R language and enriched GO and KEGG using cluster Profiler package. A total of 10 GO functions and 2 KEGG signal pathways were found which will be the main research directions in the future as shown in Figure 4 and Tables 4 and 5.

## 4. Discussion

EP is a complication of early pregnancy, and most patients will suffer from severe pelvic pain [13]. At present, the pathogenesis of EP is still unclear. Some scholars believe that embryo retention may be caused by damage to the embryo-fallopian tube environment, which leads to fallopian tube implantation [14, 15]. Pregnancy is a unique clinical situation as it can be accompanied by special diseases. Ectopic pregnancy (EP) is a complication of early pregnancy, in which the fertilized eggs are planted anywhere outside the uterine cavity without entering the uterus. Fallopian tube EP is the most common clinically. In patients' peripheral blood, it increases after treatment and is expected to become a potential observation indicator for EP treatment in the clinic. In our study, mir-196b was weakly expressed in EP patients. At present, as a research hotspot, Mir has research value in various diseases [17, 18]. We detected the miR-196b expression in peripheral blood of EP patients by qRT-PCR and found that it was significantly reduced. This suggested that miR-196b may participate in the development of EP. Moreover, we also analyzed the correlation of miR-196b with HCG and progesterone.

At present, there is relatively little research on EP and miRs. miR-196b is located on the human 7p15.2 chromosome. miR-196b has been found to have low expression in lung cancer [19], gastric cancer [20], and other tumors, but the study on EP has only been reported in the study of the team of Dominguez [12]. HCG is a glycoprotein secreted by placental trophoblast cells and consists of glycoprotein of *a* and *ß* dimers [21]. Progesterone and estradiol, as common progestins in the clinic, are important markers of EP occurrence in patients with reactions [22]. Here, through correlation analysis, we found that miR-196b is positively correlated with the expressions of HCG, progesterone, and estradiol, suggesting that miR-196b may become a potential marker of EP. Furthermore, we analyzed the changes of miR-196b in EP patients after treatment. In addition, we also found that miR-196b expression also gradually increased with the improvement of patients' therapeutic effect, which further indicates that miR-196b can be used as a potential reference indicator for observation of EP patients during treatment.

At present, the risk factors of EP are not clear clinically, but most scholars believe that pelvic inflammatory disease history, lower abdominal surgery history, abortion history, and EP history are potential risk factors of EP [23, 24]. There are relatively few clinical observation indicators after EP treatment. miR-196b expression in patients' peripheral blood after treatment was found to be increased when compared with that before treatment. In this paper, we found that miR-196b is also a potential risk factor of EP. We speculate that miR-196b plays an important regulatory role in the occurrence of EP, but its potential mechanism needs further exploration. In addition, we drew the joint ROC curve according to the indexes with different factors, and the AUC larger than 0.8 was applied to judge the potential indexes of EP.

## 5. Conclusion

At the end of the study, we predicted the potential target genes of miR-196b and analyzed its function. We found 356 potential target genes through prediction, and 10 important functions and 2 signal pathways were found through GO function enrichment, of which the RAS signal path drew our attention. The activated RAS stimulates superabundant mitotic signal cascades to promote growth and transformation cooperatively. In addition to this strong growth/transformation promoting activity, RAS also has the ability to stimulate cell apoptosis and senescence [25, 26]. Some studies have also found that RAS signal pathway is involved in the pregnancy process and has a regulatory effect [27]. This is also an important direction for our future research.

However, there are still some limitations in this study. Firstly, this study did not carry out relevant basic experiments to confirm our research conclusion. Secondly, the samples collected in this study are relatively single. Therefore, we hope to increase the number and types of our samples in future studies and carry out relevant basic experiments to verify our conclusion.

In conclusion, miR-196b is expressed in EP patients and is differentially expressed with the change of EP condition, which is expected to become a potential indicator for clinical diagnosis of EP.

## Figures and Tables

**Figure 1:** Expression of miR-196b in peripheral blood of EP patients and its correlation with HCG and progesterone. (a) qRT-PCR detected miR-196b relative expression in peripheral blood of EP patients. (b) Pearson test analyzed the correlation between miR-196b and HCG in EP patients. (c) Pearson test analyzed the correlation between miR-196b and progesterone in EP patients. (d) Pearson test analyzed the correlation between miR-196b and estradiol in EP patients. ^*∗∗∗*^*P*＜0.001.

**Figure 2:** Relationship between miR-196b changes before and after treatment of EP patients and the different therapeutic effects. (a) qRT-PCR detected miR-196b changes in peripheral blood of EP patients before and after treatment. (b) qRT-PCR detected miR-196b relative expression in peripheral blood of EP patients with different clinical curative effects after treatment. ^*∗*^*P*＜0.01; ^*∗∗∗*^*P*＜0.001.

**Figure 3:** Multivariate meaningful index combined ROC curve. When the Youden index was 68.15, the optimal specificity was 91.01%, the sensitivity was 77.14%, and the AUC was 0.899.

**Figure 4:** GO enrichment and KEGG enrichment.

**Table 1:** Comparison of baseline data between the two groups.

Factors		CG (*n* = 70)	*P* value
Age			0.444
	≥30 years (*n* = 90)	42	
	＜30 years (*n* = 69)	28	
Number of pregnancies			0.489
	Primiparity (*n* = 50)	20	
	Multipara (*n* = 109)	50	
Smoking history			0.123
	Present (*n* = 28)	16	
	Absent (*n* = 131)	54	
Place of residence			0.409
	City (*n* = 85)	40	
	Countryside (*n* = 74)	30	
Nation			0.502
	Han (*n* = 140)	63	
	Minority (*n* = 18)	7	
HCG (IU/L)		11246.97 [9172.76–12049.58]	＜0.001
Progesterone (ng/L)		25.47 [17.87–33.66]	＜0.001
Estradiol (pg/ml)		121.43 [115.32–131.19]	＜0.001

**Table 2:** Univariate analysis.

Factors		OG (*n* = 89)	CG (*n* = 70)	*P* value
History of menstrual disorder				0.598
	Present	18	12	
	Absent	70	58	
Uterine fibroids				0.502
	Present	12	7	
	Absent	77	63	
Abortion history				0.012
	Present	28	10	
	Absent	61	60	
Pelvic inflammatory disease history				0.010
	Present	25	8	
	Absent	64	62	
Lower abdominal surgery history				0.008
	Present	29	10	
	Absent	60	60	

**Table 3:** Multivariate logistic regression analysis.

Factors	*β*	S.E	Wals	Sig.	Exp (B)	EXP(B) 95% C.I.	
						Lower limit	Upper limit
Abortion history	1.811	0.619	8.563	0.003	6.114	1.818	20.56
Pelvic inflammatory disease history	1.446	0.651	4.939	0.026	4.246	1.186	15.197
Lower abdominal surgery history	1.484	0.592	6.292	0.012	4.41	1.383	14.062
miR-196b	3.639	0.537	45.9	0.000	38.06	13.282	109.069

*Note.β*: *ß* constant; S.E: standard deviation; Wals: chi-square value; Sig : *P* value; Exp (B): ratio.

**Table 4:** GO terminology.

ID	Description	*P* value	Gene ID	Count
GO:0000982	Transcription factor activity, RNA polymerase II proximal promoter sequence-specific DNA binding	3.00E-07	BACH1/EBF1/ELF4/ELK4/ERG/NR6A1/HLF/HOXA5/HOXA7/HOXB1/HOXB7/RBPJ/OTX1/PBX1/SOX11/SOX12/NR2C2/YY1/HMGA2/HAND1/TBPL1/PRDM5/ZNF281/SCRT2/FOXP2	25
GO:0000987	Proximal promoter sequence-specific DNA binding	4.04E-07	ELF4/ELK4/ERG/GATA6/NR6A1/HOXA5/HOXA7/HOXA9/HOXB1/HOXB7/RBPJ/SMAD6/OTX1/PBX1/SMARCC1/NR2C2/YY1/HMGA2/HAND1/TBPL1/ZNF516/PRDM5/ZNF281/TOX3/ZNF395/FOXP2	26
GO:0000978	RNA polymerase II proximal promoter sequence-specific DNA binding	7.50E-07	ELF4/ELK4/ERG/GATA6/NR6A1/HOXA5/HOXA7/HOXA9/HOXB1/HOXB7/RBPJ/SMAD6/OTX1/PBX1/SMARCC1/NR2C2/YY1/HMGA2/HAND1/TBPL1/PRDM5/ZNF281/TOX3/ZNF395/FOXP2	25
GO:0001077	Transcriptional activator activity, RNA polymerase II proximal promoter sequence-specific DNA binding	5.54E-06	EBF1/ELF4/ELK4/ERG/NR6A1/HLF/HOXA5/HOXA7/HOXB1/HOXB7/RBPJ/OTX1/PBX1/SOX11/SOX12/NR2C2/HMGA2/TBPL1	18
GO:0001228	Transcriptional activator activity, RNA polymerase II transcription regulatory region sequence-specific DNA binding	1.31E-05	BACH1/EBF1/ELF4/ELK4/ERG/GATA6/NR6A1/HLF/HMGA1/HOXA5/HOXA7/HOXB1/HOXB7/RBPJ/OTX1/PBX1/PBX3/SOX11/SOX12/NR2C2/HMGA2/TBPL1	22
GO:0048407	Platelet-derived growth factor binding	3.57E-05	COL1A1/COL1A2/COL3A1/PDGFRA	4
GO:0046332	SMAD binding	7.06E-05	COL1A2/COL3A1/SMAD6/TGFBR3/YY1/HMGA2/USP15/SMURF1	8
GO:0005057	Signal transducer activity, downstream of receptor	3.45E-04	CDKN1B/EPHA7/SMAD6/MAP3K1/PDGFRA/MAPK1/MAPK8/MAP4K3/FLRT1/TAOK1/NRK	11
GO:0004860	Protein kinase inhibitor activity	4.06E-04	CDKN1B/SOCS2/FLRT1/LRRC4B/SOCS4/SMCR8/SPRED1/LRRTM3	8
GO:0019210	Kinase inhibitor activity	5.36E-04	CDKN1B/SOCS2/FLRT1/LRRC4B/SOCS4/SMCR8/SPRED1/LRRTM3	8

**Table 5:** KEGG terminology.

ID	Description	*P* value	Gene ID	Count
hsa04917	Prolactin signaling pathway	2.19E-04	CCND2/NRAS/MAPK1/MAPK8/PRLR/SOCS2/SOCS4	7
hsa04014	RAS signaling pathway	2.21E-04	ABL1/ABL2/CALM1/CALM3/IGF1/NRAS/PDGFRA/MAPK1/MAPK8/RGL2/BRAP/RASGRP1/RALBP1	13

## Data Availability

The datasets used and/or analyzed during the current study are available from the corresponding author on reasonable request.
